This article has been retracted.

# Therapy Strategy of CD47 in Diffuse Large B-Cell Lymphoma (DLBCL)

**DOI:** 10.1155/2021/4894022

**Published:** 2021-09-16

**Authors:** Wenqi Zhang, Yanfeng Fan, Meng Li, Linqi Yang, Zhenya Zhang, Lihong Liu

**Affiliations:** ^1^Department of Hematology, The Fourth Hospital of Hebei Medical University, Shijiazhuang, 050000 Hebei Province, China; ^2^Department of Chemistry, Temple University, Philadelphia, Pennsylvania 19087, USA; ^3^School of Basic Medical Sciences, Hebei University of Chinese Medicine, Shijiazhuang, 050200 Hebei Province, China; ^4^Department of General Surgery, The Fourth Hospital of Hebei Medical University, Shijiazhuang, 050000 Hebei Province, China; ^5^Hebei Provincial Key Laboratory of Tumor Microenvironment and Drug Resistance, Shijiazhuang 050011, China

## Abstract

At present, the use of the common chemotherapy regimen CHOP/R-CHOP for diffuse large B-cell lymphoma (DLBCL) has some shortcomings, especially for relapsed and refractory DLBCL. CD47 is now considered as a prominent target in cancer therapies, and CD47 blockade mainly inhibits the CD47-SIRP*α* axis to prevent tumor immune escape. Here, we evaluated the effects of the latest CD47 antibodies reported and the correlations of closely related genes with CD47 in this disease. In the future, therapeutic strategies for DLBCL will focus on multitarget antibody combined treatment and multigene joint attacks.

## 1. Introduction

CD47 is a receptor that is widely expressed on the surfaces of numerous cell types and consists of *N*-terminal extracellular IgV-like domains, 5 transmembrane domains, and a short C-terminal cytoplasmic tail that functions as a transmembrane region for its immunoregulatory functions. CD47 mediates cellular phagocytosis by macrophages, the transmigration of neutrophils, and the activation of dendritic cells, T-cells, and B-cells by interacting with their ligands, including thrombospondin-1 (TSP-1), signal regulatory protein *α* (SIRP*α*), integrin, and SH2-domain bearing protein tyrosine phosphatase substrate-1 (SHPS-1). The mechanism of CD47 in tumors can be described as follows. First, CD47 is overexpressed in diverse cancers, preventing tumor cell phagocytosis and promoting tumor progression by activating the SIRP*α*-CD47 axis to thereby avoid immune surveillance. The process of macrophages phagocytosing tumor cells by blocking CD47 is demonstrated in Figure 1. Second, CD47 expression on the surface of neutrophils, dendritic cells, and T-cells inactivates immune responses to tumors by initiating reverse signaling pathways. Third, the interaction of CD47 with TSP-1 has direct anticancer and antiangiogenic effects [1]. The downregulation of CD47 expression may induce the removal of aged and superfluous cells through phagocytosis, which plays a crucial role in various homeostatic systems [2]. However, the role of CD47 in several malignant tumors, including hematological malignancies, such as leukemia, lymphoma, and multiple myeloma, has been assessed in many studies. This molecule is expressed at varying levels on a variety of hematopoietic and nonhematopoietic cells. Most cancer cells overexpress CD47, and its expression level independently correlates with poor clinical outcomes in patients with hematological and solid tumor malignancies [3, 4].

Diffuse large B-cell lymphoma (DLBCL) is the most common aggressive lymphoid malignancy, and rituximab, cyclophosphamide, doxorubicin, and prednisone (R-CHOP) therapy is one of the most effective treatment strategies for most DLBCL subtypes [5]. Currently, CHOP and R-CHOP are the most widely used chemotherapies for DLBCL. Patients with DLBCL who become resistant to standard chemotherapies and antibody-based regimens or relapse might have poor prognoses. Approximately 40% of patients treated with R-CHOP die after developing intrinsic resistance or relapsing. Unlike the limited effects of single-drug therapies for DLBCL, combination therapies were suggested to yield good treatment responses in several studies. As a promising immunomodulatory therapeutic strategy, blockade of CD47 has been evaluated in early clinical trials. High CD47 mRNA expression was correlated with the poor survival of DLBCL patients, highlighting DLBCL as a candidate for future CD47-targeted therapies. This review focuses on the latest studies on DLBCL treatments related to CD47.

## 2. Applications of CD47 in Clinical Therapies

SIRP*α* and TSP-1 are the two most important endogenous ligands of CD47. SIRP*α* is expressed on the plasma membranes of all myeloid and neuronal cells as a transmembrane glycoprotein [6]. The CD47-SIRP*α* axis plays a crucial role in tumor development. CD47 acts as a “do not eat me” receptor by interacting with SIRP*α* on the healthy macrophage surface membrane and prevents phagocytosis by triggering a dephosphorylation cascade [7–9]. Vascular growth factor (VEGF) and its receptor (VEGFR2) can be activated by TSP-1 and CD47 in combination to stimulate angiogenesis, and the interaction between CD47 and integrin *α*V*β*3 enhances neovascularization to allow tumor growth [10]. Studies have shown that the overall survival (OS) and progression-free survival (PFS) of DLBCL patients, especially those with the activated B-cell-like (ABC) subtype, are significantly reduced when both CD47 on tumor cells and SIRP*α* in stromal cells are upregulated or when only SIRP*α* expression is increased. In an *in vitro* study of bone marrow-derived macrophages, the interaction between CD47 and SIRP*α* polarized macrophages toward an M2 immunosuppressive phenotype, which provided an abundant tumor-associated macrophage (TAM) microenvironment [11]. This result indicated that tumor cells and stromal cells might interact with each other, worsening the prognoses of patients. As the combined expression of CD47 and SIRP*α* is potentially an independent prognostic factor for DLBCL, the levels of CD47 and SIRP*α* before CD47 blockade therapy need to be evaluated [12].

Previous studies reported that calreticulin and phosphatidylserine could induce phagocytosis by binding to the low-density lipoprotein receptor-associated protein (LRP) on phagocytes, as blocking the CD47-SIRP*α* antiphagocytic signal induced an effective prophagocytic signal to trigger tumor phagocytosis [13, 14]. In humans, calreticulin is commonly expressed at higher levels in the cells of several hematological malignancies, including non-Hodgkin's lymphoma (NHL), than in normal bone marrow and peripheral blood cells. In addition to interfering with the SIRP*α*-CD47 interaction, CD47 antibodies can cause tumor-specific T-cell reactions, such as CD8+ cell activations [15]. Functional CD47 antibody blockades could be targeted to tumor stem cells to promote radiotherapy sensitivity in tumors and protect normal tissues [16–19].

Treatment with 9-cis-retinoic acid and interferon *α* (RA/IFN-*α*) triggers early membrane exposure to calreticulin, the expression of heat shock proteins (HSPs) 70 and 90, the downregulation of CD47 expression, and the enhancement of HMGB1 secretion [20]. This drug was shown to upregulate the expression of the NOXA protein in DOHH2 DLBCL cell lines to induce a strong apoptotic response [21, 22]. This study provides a new approach for dendritic cell (DC) immunotherapies based on therapeutically relevant immunogenic cell death (ICD) for relapsed and/or refractory (R/R) lymphoma, which promotes intense antitumor responses by inducing Th1 immunity [23–25].

## 3. Preclinical Trials on CD47 Antibodies

As shown in preclinical studies, anti-CD47 antibodies can be used in combination. In current clinical trials, four different antibody molecules designed to target CD47-SIRP*α*, Hu5F9-G4, CC-90002, TTI-621, and ALX-148 are being assessed for their ability to treat malignant tumors. Among them, Hu5F9-G4 and TTI-621 were demonstrated to effectively treat DLBCL in several studies [26].

### 3.1. Hu5F9-G4

Hu5F9-G4 (hereafter, 5F9), an anti-CD47 humanized IgG4 antibody that binds to monomeric human CD47, is currently being assessed in four different phase I trials and has received fast-track designation by the US Food and Drug Administration for further development for the treatment of DLBCL and follicular lymphoma (FL). Treatment with 5F9 induces macrophages to recognize and attack cancer cells by preventing the activation of the CD47-SIRP*α* axis and promoting the phagocytosis of tumor cells via innate immune cells [1, 27].

Moreover, 5F9 was shown to augment the activity of rituximab (Rituxan; Genentech) and to synergistically affect lymphoma in preclinical models. A recent phase 1b trial involving heavily pretreated patients with R/RDLBCL and FL indicated that the combination of 5F9 and rituximab (NCT02953509) induced a high rate of tolerable and durable complete responses. This combination therapy resulted in a 40% overall response (OR) and a 33% complete response (CR) in R/R DLBCL patients. However, the objective response rate achieved with this treatment was higher for patients with ABC-DLBCL than GCB-DLBCL (67% for ABC-DLBCL vs. 17% for GCB-DLBCL) [28].

Moreover, 5F9 was recently assessed in a first-in-human phase I trial on patients with advanced solid tumors and lymphomas to evaluate its safety, pharmacokinetics (PK), and pharmacodynamics. The trial showed that 5F9 was well tolerated at a priming dose of 1 mg/kg on day 1 and maintenance dose of up to 45 mg/kg weekly. A linear PK curve was observed for 5F9 doses exceeding 10 mg/kg. In regard to saturating concentrations, the agent was administered biweekly and had a terminal half-life of approximately 13 days. The most common drug-related adverse event (AE) resulting from 5F9 treatment was expected, on-target, mild, transient, and predictable anemia which was mitigated by administering priming and maintenance doses in cycle 1. As younger red blood cells (RBCs) lack prophagocytic signals, older RBCs were perturbed by CD47 blockade in most cases. To circumvent the hemolytic anemia and thrombocytopenia caused by the expression of CD47 on red blood cells and platelets, different strategies, such as newly developed BsAbs and priming with low-dose levels to eliminate aging RBCs, are being investigated. Additional clinical trials are required to assess the clinical efficacies of these strategies.

At doses of 20 mg/kg and higher, chills, headache, fatigue, and fever were frequently observed, with most occurring within the first cycle of grade 1 or 2. Pretreatment with acetaminophen and diphenhydramine before the first two doses of 5F9 was recommended to decrease the incidence and severity of these side effects. Abdominal, back, and chest pain in a few patients during infusion were not related to other clinical findings. Temporarily stopping or slowing the rate of infusion often mitigated these effects. Nevertheless, dose-related thrombocytopenia and neutropenia were not observed. Thus, 5F9 might be readily combined with other antitumor antibodies according to this favorable safety assessment.

Due to the mild and manageable 5F9-related AEs and easy administration of 5F9 infusions in an outpatient setting, this treatment might be beneficial in older patients with aggressive and relapsed lymphomas who cannot tolerate other treatments [27, 29, 30].

### 3.2. TTI-621

As a novel checkpoint inhibitor, TTI-621 (SIRP*α*-IgG1 Fc) is a soluble, fully human recombinant fusion protein designed to block the CD47 “do not eat me” signal by IFN primed macrophages that triggers tumor cell phagocytosis. TTI-622 is another SIRP*α* Fc decoy receptor under investigation for anticancer treatment. Although they have very similar effects, most studies have focused on TTI-621 [1].

TTI-621 could improve the treatment toleration of R/R DLBCL patients. Moreover, TTI-621 effectively induced the destruction of cancer cells by various sets of TAMs and the phagocytosis of lymphoma cells by all macrophage subtypes in vivo. TTI-621 has a synergistic effect on the phagocytosis of tumor cells mediated by FC *γ* r CD64 and CD32. Early results from an *in vitro* study showed that M (-), M (IL-4), and M (HAGG+IL-1 *β*) macrophages had a slightly worse phagocytic response to TTI-621 than the M (IFN-*γ*+-LPS) and M (IL-10+TGF *β*) subtypes. Cytokines (IFN-*γ*, IFN-*α*, or IL-10) or TLR agonists (LPS, poly (I: C) or R848) could easily repolarize these cells into highly phagocytic macrophages [31].

TLR-3, TLR-4, and TLR-7 synergize with CD47 blockade on tumor cells by enhancing secretion and exposing calreticulin on the macrophage surface in a Btk-dependent manner [32]. TTI-621 and TLR agonists in combination are a potential strategy for the treatment of hematological malignancies in the future (NCT02663518).

The safety and activity of TTI-621 in R/R hematologic malignancies were evaluated in a first-in-human phase I study (NCT02663518). Among evaluable patients with DLBCL, 23% had objective responses, including 29% patients who received TTI-621 monotherapy and 21% patients who received TTI-621 combination therapy with rituximab (0.1 mg/kg). The median overall response time of DLBCL patients was 78 days, and the median treatment duration was 143 days. The observed activity suggests that TTI-621 can be used as a monotherapy. Combination with a second agent to elicit the necessary prophagocytic signal is not required, since TTI-621 provides adequate intrinsic activation signals and active Fc regions. The clinical efficacy of TTI-621 is better than those of anti-CD47 agents with less active Fc regions, such as Ig4-based molecules (5F9). The next stage of this ongoing study is to determine the recommended dose of TTI-621 in phase II trial.

The most common side effects of TTI-621 during treatment were infusion-related reactions (43%), thrombocytopenia (26%), chills (18%), fatigue (15%), anemia (13%), nausea (12%), pyrexia (10%), and diarrhea (10%). Infusion-related treatment reactions usually occurred after the first dose and were rarely grade 3 or higher. The incidence of treatment-related anemia for any grade was 13%, and 9% of patients had anemia of grade 3, which was lower than that of a phase I study on 5F9. Treatment-related anemia occurred in 41% of patients with R/R NHL treated with TTI-621 combined with rituximab, and most of them were grade 3 [28].

In contrast with 5F9, the use of an anemia-mitigating priming dose regimen is not required for anemia caused by TTI-621. Both TTI-621 and TTI-622 exhibit minimal binding to human red blood cells. Compared to those treated with 5F9, patients treated with TTI-621 and TTI-662 have a lower risk of anemia during treatment. However, 20% of subjects receiving TTI-621 exhibited treatment-related thrombocytopenia of grade 3 or higher, which was higher than that of 5F9 (5%), and this percentage did not increase as the dose increased. Nevertheless, this effect was reversible, and the patients recovered within 1 week without severe bleeding or dosing interruptions. Overall, TTI-621 is promising as both a monotherapy and in combination [33].

### 3.3. NI-1701

NI-1701 is a new high-affinity fully human bispecific antibody (biAb) designed to selectively coengage CD47 and CD19 on B-cells to maximally inhibit tumor growth by phagocytosing the targeted cells. NI-1701 is a *κλ*-body consisting of a high-affinity CD19 targeting arm and an appropriate CD47 blocking arm on a human IgG1 Fc backbone [34, 35]. The Fc domain of anti-CD47 monoclonal antibodies, such as IgG4 (5F9), has been selected to weaken effector functions. Mediated by Fc, this function can prevent CD47 targeted monoclonal antibodies from selectively eliminating healthy host cells. However, this function limits tumor lethality as a monotherapy at the same time. NI-1701 has an Fc-mediated full spectrum effector function. The combination of a high-affinity CD19 binding arm and a low-affinity CD47 arm could highly expand the safety range of CD47-targeted therapies [36]. Therefore, this treatment shows favorable elimination kinetics and overcomes the limitations of other CD47-targeted agents, such as rapid drug elimination and hemotoxicity which can significantly shift the signal for binding to only B-cells and weakly binding to platelets, T-cells, and erythrocytes. ACD47 mAb (hB6H12) could combine with all cells as a control group for CD47 expression. The final tumor growth inhibition (TGI) of NI-1701 was 79%, which was substantially better for controlling tumor growth than rituximab, with a TGI of 48%. NI-1701 also slowed tumor growth for a longer period. Interestingly, NI-1701 and rituximab in combination had a higher TGI (92%) at the end of the treatment period. The survival time was increased by 2.45-fold for patients treated with the two drugs in combination (60 days in the combined treatment group compared to 24.5 days in the control group) [37]. The comparison between Hu5F9-G4, TTI-621, and NI-1701 is listed in Table 1.

## 4. Crosstalk between CD47 and Other Genes

Studies and bioinformatics analyses have demonstrated that CD47 is associated with other DLBCL-related genes, such as PD-L1, LAG-3, TIM-3, and CD4.

### 4.1. PD-L1

Cancer cells utilize the programmed cell death 1/programmed cell death ligand 1 (PD-1/PD-L1) pathway to suppress immune cells (including T-cells, B-cells, natural killer cells, lymphocytes, and dendritic cells), leading to poor prognoses in various cancers. As a predictive biomarker, PD-L1 is better used in anticancer monotherapy than combination therapies [38]. PD-1/PD-L1 inhibitors can restore T-cells and improve antitumor immune responses. A clinical study of 121 DLBCL patients showed that immune chemotherapy lowered the levels of soluble PD-1 (sPD-1), and high pretreatment PD-1 levels were associated with poor clinical outcomes. PD-1 is a predictor of the histological transformation (HT) of FL to DLBCL [39–43]. In primary central nervous system diffuse large B-cell lymphoma (PCNS-DLBCL), the PD-1/PD-L1 signaling pathway plays an important role in the immune microenvironment, which correlates with increased sensitivity to chemotherapy and OS. Both PD-1 and PD-L1 are expressed on TILs and tumor cells.

The overexpression of PD-L1 in tumor B-cells was shown to be significantly associated with PD-1 in TILs, and patients with high PD-1 levels in TILs have low survival rates. Epstein–Barr virus (EBV) may be affected by lymphoma cells in posttransplant lymphoma proliferative disorder (PTLD) due to immune surveillance escape.

PD-L1 was reported to be overexpressed in 60% of PTLD patients in immunodeficiency states, and the EBV induced PD-L1 expression in TAMs. A study on 273 patients showed that the upregulation of PD-L1 and mPD-L1 expression in DLBCL cells was significantly associated with non-GCB type and EBV positively, and these patients had a lower OS than DLBCL patients with downregulated PD-L1 expression [41, 44, 45].

### 4.2. LAG-3

Lymphocyte activation gene-3 (LAG-3, CD223) belongs to the immunoglobulin superfamily and plays a negative regulatory role in T-cell homeostasis. The upregulation of LAG-3 expression was first discovered in activated CD4+, CD8+, and NK cell subsets, but this molecule was also shown to be highly expressed on Treg27 cells as an immunosuppressive molecule.

LAG-3 can be activated upon binding to major histocompatibility (MHC) class II molecules, inhibiting the activity of T lymphocytes and eventually leading to T-cell anergy. A set of genes in cancer immune evasion pathways (immune escape gene set, IEGS) includes TIMP1, LGALS3, CCL2, IL6ST, LGALS1, CD163, IDO1, VEGFA, CSF1, IL-10, LAG-3, MRC1, CTLA4, CD274 (PDCD1LG1), TIGIT, SOCS3, PDCD1LG2, PVR, HGF, GDF15, IDO2, HAVCR2, MSR1, JAK2, LAIR1, CCL22, MCL1, PDCD1, and PIM1 (*p* values from 5.10^−12^ to 3.10^−2^). The IEGS gene sets were highly enhanced in DLBCL cells compared to normal B-cells. The LAG-3 gene was upregulated by 3.4-fold in DLBCL cells relative to the control groups (*p* < 10^−13^), and LAG-3 might promote tumor escape in DLBCL [42].

### 4.3. TIM-3

T-cell immunoglobulin and mucin domain-containing protein-3 (TIM-3, HAVCR2) is a type I transmembrane protein that is most notably expressed on CD4+ Th1 and CD8+ cytotoxic T-cells to limit the duration and magnitude of T-cell responses. TIM-3 is encoded by HAVCR2, which is located on human chromosome 5. TIM-3 is comprised of 301 amino acids, and its structure includes four regions: an extracellular IgV domain, a mucin domain, a transmembrane region, and a cytoplasmic tail.

Immunohistochemistry analysis of tumor cells and TIL samples from 123 untreated DLBCL patients indicated that TIM-3 was highly expressed in DLBCL tumor cells, and more than one-third of patients (39%) also exhibited TIM-3 expression in TILs. In univariate analysis by controlling for the international prognostic index (IPI) score, a correlation was observed between TIM-3 overexpression and poor OS, resulting in decreased immune surveillance and tumor clearance, was reported [43]. TIM-3 is also highly expressed in peripheral blood CD3+ T-cells from patients with DLBCL and is related to tumor stage and responses to conventional chemotherapy [46, 47].

LAG-3 and TIM are associated. In an EBV-DLBCL study, the Colm Keane research group performed EBV-encoded small RNA in situ hybridization, and the results were digitally quantified (EBER-digital) in 390 cases, comparing the host gene expression results, stratified by the EBER-digital status. Strong associations were observed among immune-related genes in EBV-positive tumors. The immune checkpoints PD-L1 (*p* < 0.0001), PD-L2 (*p* = 0.08), LAG-3 (*p* = 0.01), and TIM-3 (*p* = 0.05) were expressed at higher levels in EBV-positive patients than in EBV-negative patients, and the EBV-negative biopsies revealed similar results. In EBV-DLBCL, LAG-3 and TIM-3 might interact to balance the high level of immunosuppression in the tumor microenvironment (TME) with the increased level of immune checkpoints and tumor-associated macrophages, thus affecting the survival rate [48].

### 4.4. CD4

CD4 expression serves as a T-cell marker, and its expression in DLBCL is rare and aberrant. Under normal circumstances, T-cell antigens are not abnormally expressed in B-cell lymphoma, and only 10 cases of CD4+ DLBCL have been reported thus far. ALK- CD4+ was observed in all ten cases, including nine cases of DLBCL and one case of primary mediastinal large B-cell lymphoma (PMLBCL) [49].

The density of CD4+ lymphoma cells was increased among ALK+ DLBCL patients. However, CD4 is rarely expressed in DLBCL, not otherwise specified (NOS), with only 4 cases being reported worldwide. This intriguing phenomenon raises questions regarding lineage fidelity and the biology underlying such unusual expression. A few hypotheses have been proposed to explain this phenomenon: for example, the dysregulation of malignant B-cell gene expression may lead to the activation of other silenced or inhibited T-cell differentiation genes, and tumors may cause abnormal expression at the stem cell level. Although the mechanism and importance of this phenomenon are currently uncertain, it leads to interesting biological and diagnostic considerations.

#### 4.4.1. Data Source

The study was carried out using these two strategies and several steps. The data shown in graphs (a) through (d) in Figure 2 were obtained from the GEPIA database (http://gepia.cancer-pku.cn/detail.php). This dataset was selected from DLBCL tumor cells. The Pearson correlation coefficients were calculated on a nonlog scale, and the log-scale axis was used for visualization. The target genes of Figure 2(e) were identified from the whole-genome expression data of human lymphoblast cells found on the GeneNetwork website (http://www.genenetwork.org/webqtl/main.py). This dataset was produced by using lymphoblast B-cell mRNA from UTHSC CEPH B-cells Illumina (Sep09) RankInv. Because GEPIA and the gene network data sources differ, DLBCL tumor cells were not collected from the GeneNetwork database, and the results from these two platforms might thus be slightly biased [50].

### 4.5. GEPIA Correlation Analysis

In DLBCL, CD47 was positively correlated with TIM-3, LAG-3, and CD4, among which the correlation between CD47 and LAG-3 was the strongest (*r* = 0.68), and CD47 and PD-L1 had the weakest correlation (*r* = 0.32). The *R* value of CD47 and TIM-3 was 0.51, and that of CD47 and CD4 was 0.58. All of the correlation coefficients of CD47 with other genes, except for PD-L1, were greater than 0.5, indicating that they were closely related.

### 4.6. QTL Mapping of Four Gene Probes

Since CD4 was not associated with the other four genes after several *R* values were adjusted, only the remaining four genes in the QTL analysis will be discussed. The expression data from only one of CD47, LAG-3, TIM-3 (HAVCR2), and PD-L1 (CD274) probes were extracted from the human lymphoblastoid cell database. In Figure 2(e), CD47 was shown to be directly related to LAG-3 and TIM-3, while PD-L1 was directly connected to LAG-3, thus indicating an indirect relationship with CD47. The *R* value of CD47 and TIM-3 was 0.48, suggesting the strongest and most positive correlation, while the absolute value of CD47 and LAG-3 was 0.35 and negatively correlated. In the QTL data analysis, CD47 and TIM-3 had the closest relationship among the four genes. However, CD47 and PD-L1 were not related, with a low *R* value of 0.03. The *R* value of PD-L1 and LAG-3 was 0.36, demonstrating a positive correlation.

Although no direct correlation between CD47 and PD-L1 in DLBCL has been reported to date, they both undeniably play important roles in DLBCL, and their “do not eat me” and “do not find me” signaling relationship is essentially interesting. While these two genes did not have a high correlation value, a strong correlation was observed between LAG-3 and CD47, indicating that CD47 and PD-L1 might be linked through LAG-3 via other potential pathways.

TIM-3 and LAG-3 are the most frequently reported genes in DLBCL among these four genes, and they are also closely related to CD47 as immune checkpoints. Moreover, CD47 exhibited direct relationships with TIM-3 and LAG-3, which indicates the potential and value of a follow-up study on the interactions among CD47, LAG-3, and TIM-3 in DLBCL.

The expression of CD4 in DLBCL is an unexpected phenomenon. Interestingly, CD47 and CD4 were strongly correlated in the GEPIA analysis. Although the mechanism by which CD4 functions as a T-cell antigen in DLBCL remains unclear and there are no reports of this molecule interacting with CD47 in this disease, these findings can be used as a reference for further studies on the role of CD4 in DLBCL.

## 5. Conclusion and Future Perspectives

In conclusion, CD47 is a potential target for the treatment of DLBCL, especially for relapsed and refractory DLBCL. Treatment strategies include multitarget combination therapies, such as CD47 monoclonal antibodies combined with CD20 and CD19. The emerging antibodies TTI-621 and NI-1701 were not limited by the adverse reactions of Hu5F9-G4, such as anemia, and showed better therapeutic effects. Moreover, CD47 was highly associated with TIM-3 and LAG-3 in DLBCL at the gene level. Additionally, PD-L1 is a checkpoint commonly used for targeted hematological cancer therapies, and PD-L1 and CD47 in combination have attracted increased attention. A pathway involving CD47 and these genes may exist in this disease, which needs to be verified in ongoing clinical studies to provide new insights for future DLBCL treatment strategies.

## Figures and Tables

**Figure 1:** Blocking CD47 induces the phagocytosis of tumor cells by macrophages.

**Figure 2:** The quantitative trait locus (QTL) mapping and GEPIA correlation analysis of CD47 with Programmed Death-Ligand 1(PD-L1, CD274), lymphocyte activation gene-3 (LAG-3), T-cell immunoglobulin and mucin domain-containing protein-3 (TIM-3, HAVCR2), and CD4. (a) Positive correlation between LAG-3 and CD47 probes. (b) Positive correlation between TIM-3 (HAVCR2) and CD47 probes. (c) Positive correlation between CD4 and CD47 probes. (d) Positive correlation between PD-L1 (CD274) and CD47 probes. (e) The 4 nodes in the network graphs display the 3 traits among the CD47 (1771333), PD-L1 (1794040, CD274), LAG-3 (1813338), and TIM-3 (1693826, HAVCR2) genes. Only Pearson correlation coefficients greater than 0.35 or less than −0.35 are shown.

**Table 1:** The comparison of anti-CD47 antibodies for treatment of DLBCL.

Name	Hu5F9-G4	TTI-621	NI-1701
Characteristic	Monoclonal antibody	Fusion protein	Bispecific antibody
Target	CD47	CD47 SIRP*α*	CD47 CD19
Phase	Phase I/II clinical	Phase I clinical	Phase I clinical
IgG subclass	IgG4	IgG1	Engineered IgG1
AEs	Anemia, thrombocytopenia ≥ 20 mg/kg: chills, headache fatigue, fever	Infusion-related reactions, thrombocytopenia, chills, fatigue, anemia, nausea, pyrexia, diarrhea	
